# Transdermal nitroglycerine enhances postoperative analgesia of intrathecal neostigmine following abdominal hysterectomies

**DOI:** 10.4103/0019-5049.60492

**Published:** 2010

**Authors:** Fareed Ahmed, Ashish Garg, Vipul Chawla, Mamta Khandelwal

**Affiliations:** Department of Anaesthesia and Critical Care, Sawai Man Singh Medical College and Hospital, Jaipur - 302 004, Rajasthan, India

**Keywords:** Abdominal hysterectomy, neostigmine, nitroglycerine, nitric oxide, postoperative analgesia

## Abstract

This study was carried out to assess the effect of nitroglycerine (transdermal) on intrathecal neostigmine with bupivacaine on postoperative analgesia and note the incidence of adverse effects, if any. After taking informed consent, 120 patients of ASA Grade I and II were systematically randomised into four groups of 30 each. Patients were premedicated with midazolam 0.05 mg/kg intravenously and hydration with Ringer's lactate solution 10ml/kg preoperatively in the holding room. Group I patients received Intrathecal injection of 15 mg bupivacaine with 1ml of normal saline and transdermal placebo patch. Group II patients received Intrathecal injection of 15 mg bupivacaine with 5 mcg of neostigmine and transdermal placebo patch. Group III patients received Intrathecal injection of 15 mg bupivacaine with 1ml of normal saline with transdermal nitroglycerine patch (5 mg/24 hours). Group IV patients received Intrathecal injection of 15 mg bupivacaine with 5mcg of neostigmine and transdermal nitroglycerine patch (5 mg/24 hours), applied on a non anaesthetised area after 20 minutes. Groups were demographically similar and did not differ in intraoperative characteristics like sensory block, motor block, haemodynamic parameters and SpO_2_. The mean duration of analgesia was 202.17 minutes, 407.20 minutes, 207.53 minutes and 581.63 minutes in control group (I), neostigmine group (II), nitroglycerine group (III) and nitroglycerine neostigmine group (IV) respectively (P<0.01). To conclude, our results show that transdermal nitroglycerine itself does not show any analgesic potential but it enhances the analgesic potential of intrathecal neostigmine.

## INTRODUCTION

Nitric oxide (NO) has been suggested to act as a second messenger in the central nervous system (CNS)[1–4] and has been shown to play an important role in the mechanisms that underlie pain.[5–7] NO, produced from L-arginine by NO synthase,[8,9] produces an increase in intracellular cyclic GMP (cGMP) through activation of soluble guanylate cyclase. This NO-cGMP cascade in endothelial cells has been reported to mediate acetylcholine-induced vasodilation[4,10] as well as to be involved in acetylcholine or morphine induced antinociception.[11,12] Therefore, as acetylcholine-induced responses have been shown to involve NO, the present experiments were designed to examine whether a combination of transdermal nitroglycerine (source of exogenous nitric oxide) would enhance the analgesic efficacy of intrathecal neostigmine (source of acetylcholine) in patients undergoing abdominal hysterectomy. There is paucity of work done involving humans subjects.

## METHODS

This prospective, randomised, double blind study was approved by the Ethical Committee of Rajasthan University of Health Sciences, Jaipur. After taking informed consent, 120 patients of ASA Grade I and II, aged between 30 to 50 years, scheduled for elective total abdominal hysterectomy were selected.

A total of 126 patients were selected for the study. Six patients were excluded because of failed/partial spinal block (effective sample size *n* =120). The principles of simple randomisation were applied. Patients were randomised by computer into one of the four groups consisting of 30 patients in each group and prospectively studied.

Group I patients received 3 ml (15 mg) of hyperbaric bupivacaine (0.5%) plus 1 ml normal saline with transdermal placebo patch. Group II patients received 3 ml (15 mg) of hyperbaric bupivacaine (0.5%) plus 5mcg neostigmine and transdermal placebo patch. Group III received 3 ml (15 mg) of hyperbaric bupivacaine (0.5%) plus 1 ml normal saline and transdermal nitroglycerine patch (5 mg/24 hours). Group IV received 3 ml (15 mg) of hyperbaric bupivacaine (0.5%) plus 5 mcg neostigmine and transdermal nitroglycerine patch (5 mg/24 hours).

In the preanaesthesia room, patients were premedicated with midazolam 0.05 mg/kg IV and preloaded with crystalloid 10 ml/kg. Inside the operation theatre, lumbar puncture was performed at L3-L4 level, with 25 gauge spinal needle and 4 ml of the drug solution was injected intrathecally over 30 seconds as per the group allocation. They were then placed in supine position, with a 15° head low tilt immediately after spinal injection. An eye cover was placed and O_2_ was given by Hudson mask at the rate of 4 L/min by the anaesthesia machine. The transdermal patch (placebo or nitroglycerine) was applied on the thorax (ventral, T2-T4), in a non-anaesthetised area, 20 minutes after spinal puncture (after haemodynamic stabilisation). The total nitroglycerin content of transdermal nitroglycerine patch was 25 mg; the total drug releasing area was 10 cm^2^. It delivered nitroglycerine at the rate of 20-25 *μ*g/cm^2^.h or. 5 mg/24 hours.

The drug solution was prepared by the anaesthesiologist who performed the lumbar puncture, administered the drug solution and monitored the patient intraoperatively. Patients were evaluated for postoperative analgesia and adverse effects by another anaesthesiologist blinded to the drug groups.

Level of sensory loss was assessed by pinprick test. Motor blockade was determined according to the Bromage scale. Blood pressure was monitored every five minutes throughout the surgery and a decrease greater than 15% below the baseline value was treated by the incremental dose of Injection ephedrine 4 mg IV. Heart rate and SpO_2_ were monitored continuously. Any fall in the heart rate below 60 beats per minute was treated with incremental doses of Inj. atropine 0.3 mg IV. Intraoperative nausea was treated with Inj. metaclopromide 10 mg intravenous.

All patients were familiarised with 0-10 cm visual analogue scale, for pain (VAS); 0 equal to “no pain” and 10 equal to “worst possible pain”. VAS was assessed at the time of giving rescue analgesia. Postoperatively, patients were assessed for pain by VAS rating scale and duration of motor blockage according to the Bromage scale. Patients were also assessed for the side-effects like nausea, vomiting, hypotension, bradycardia, sweating and palpitation.

Duration of effective analgesia was measured from the time of intrathecal drug administration to the patient's first request for analgesic. Patients were allowed to receive rescue analgesics on demand. Intramuscular Diclofenac (75 mg) was given as rescue analgesic. Groups were compared with regard to demographic data (age, weight), duration of surgery and duration of analgesia with use of one-way analysis of variance. *P* value <0.05 was considered statistically significant.

## RESULTS

There was no statistically significant (*P*>0.5) difference among all four groups in terms of demographic data, type and duration of surgery and changes in the haemodynamic parameters [Table 1]. The onset of sensory block, measured by pinprick was 6.23±1.65, 3.13±0.90, 5.80±1.75 and 3.27±0.83 minutes in Group I, II, III and IV respectively [Table 2]. Onset of sensory block was faster (statistically significant) in neostigmine using groups (Group II, IV) *c.f.* non-neostigmine using groups (Group I, III) (*P*<0.05) [Table 2]. The mean duration of analgesia was 202.17 minutes, 407.20 minutes and 207.53 minutes in control group (I), neostigmine group (II) and nitroglycerine group (III) respectively, while the mean duration of analgesia in nitroglycerine neostigmine group (IV) was 581.63 minutes [Table 2]. A statistically significant longer duration of analgesia in Group IV was observed when compared to Group II (*P*<0.01). The onset of motor block was 12.47±2.78 minutes and 11.17±2.76 minutes in Group I and III while it was 5.47±1.04 and 5.33±1.09 minutes in Group II and IV (*P*<0.05) [Table 2]. The mean duration of motor block was 79.77±6.73, 102.87±5.99, 77.77±5.26 and 103.13±6.14 minutes in Group I, II, III and IV respectively [Table 2]. The average VAS pain score at the time of giving rescue analgesic medication was 22.81±7.29, similar among all four groups (P>0.05). Table 3 shows the haemodynamic parameters i.e. mean arterial pressure (MAP), pulse rate (PR) during the preoperative, intraoperative and postoperative period. The incidence of side-effects seen in all four groups is shown in Table 4.

**Table 1:** Demographic profile of groups with mean and S.D values

	Group I	Group II	Group III	Group IV
Number of patients	30	30	30	30
ASA grade (I/II)	16/14	13/17	19/11	17/13
Age (Yrs)*	39.57±5.44	38.97±6.14	41.30±5.29	39.90±5.73
Weight (Kg)*	54.03±5.54	51.57±6.95	50.57±3.35	53.03±6.23
Surgical time (min)*	65.50±9.86	63.50±10.01	65.17±9.96	63.50±11.61

* *P*>0.05 (Non-Significant)

**Table 2:** Onset, duration of analgesia and relaxation (mean ± s.d)

Group	Onset in minutes		Duration in minutes	
		
	Sensory block	Motor block	Analgesia	Relaxation
I	6.23±1.65	12.47±2.78	202.17±18.23	79.77±6.73
II	3.13±0.90	5.47±1.04	407.20±53.21	102.87±5.99
III	5.80±1.75	11.17±2.76	207.53±16.33	77.77±5.26
IV	3.27±0.83	5.33±1.09	581.63±64.93	103.13±6.14

**Table 3:** Haemodynamic parameters (mean± s.d)

Group	Pre-operative		Intra-operative		Post-operative	
			
	MAP	PR	MAP	PR	MAP	PR
I	94.67±8.64	84.67±8.59	89.03±4.64	82.77±11.22	89.71±3.92	86.93±4.28
II	93.65±6.46	84.83±11.65	85.35±8.07	83.33±8.64	89.07±4.14	86.83±8.68
III	92.55±5.97	88.30±8.15	86.08±7.32	83.60±7.47	93.99±6.33	80.00±7.59
IV	94.00±8.49	85.77±9.60	90.67±7.56	82.70±9.12	86.48±6.23	78.63±9.20

MAP: Mean arterial pressure in mm Hg, PR: Pulse rate

**Table 4:** Side-effects and complications

Groups	Nausea		Vomiting		Sweating		Hypotension		Bradycardia	
					
	No.	%	No.	%	No.	%	No.	%	No.	%
I	3	10	2	6	-	-	5	15	1	3
II	2	6	2	6	1	3	1	3	1	3
III	3	10	2	6	-	-	3	10	-	-
IV	2	6	2	6	1	3	1	3	-	-

## DISCUSSION

In clinical practice, a number of adjuvant have been added to the intrathecal local anaesthetics for supplementation of intraoperative anaesthesia and postoperative analgesia. They have advantages as they reduce the dose of local anaesthetic; provide long lasting postoperative analgesia with reduced incidence of central nervous system depression, motor effects or hypotension.

The results of this study show a significant increase in postoperative analgesia when neostigmine is added to intrathecal bupivacaine in patients undergoing total abdominal hysterectomy. Neostigmine-induced augmentation of analgesia, when supplemented to bupivacaine, has been shown in other studies.[13–15] Further, the present study showed that the combination of 5 mg/day transdermal nitroglycerine patch and intrathecal low dose neostigmine (5 mcg) resulted in an average of 10 hours of postoperative analgesia after total abdominal hysterectomy during bupivacaine spinal block, compared to 3.5 hours in the control group. The combination increased the duration of analgesia, as the first requirement of rescue analgesia was delayed by 6.5 hours in this group compared from the control group. In a similar study, authors observed that intrathecal neostigmine along with transdermal nitroglycerine patch provided longer duration of analgesia and significantly minimized the analgesic consumption than only intrathecal neostigmine.[16] Another worker reported 6.50 hours of analgesia in neostigmine group, compared to 9.10 hours of analgesia in nitroglycerine-neostigmine group.[14] Transdermal nitroglycerine has been shown to increase the postoperative analgesia of intrathecal opioids.[17] Our study demonstrates no clinically significant difference in the haemodynamic parameters and adverse effects among all four groups. Similarly, a study reported no increase in adverse effects using intrathecal neostigmine with transdermal nitro-glycerine.[16] Intrathecal neostigmine doses varying from 10 mcg to 200 mcg resulted in side-effects (namely, nausea and vomiting) when doses varied between 25 and 200 mcg.[18,19]

Analgesic effect of intrathecal neostigmine is secondary to acetylcholine release in the spinal cord tissue.[20,21] During surgical stimuli, a pre-existent spinal cholinergic tonus is activated.[22] Neostigmine, an anticholinsterase drug increases the concentration of acetylcholine in the cerebrospinal fluid and acetylcholine bioavailability at the cholinergic nerves within the spinal cord. Elevated acetylcholine due to the surgical stimulus and also acetylcholine preserved from cholinesterase activity after intrathecal neostigmine, binds to muscarinic[23] and nicotinic[24] nerve terminals in the spinal cord.

The existence of a cholinergic system in the spinal dorsal horn involved in sensory transmission and modulation is supported by anatomical, pharmacological and electrophysiological studies. For example, Choline Acetyltransferase (ChAT)-positive terminals are found in the spinal dorsal horn[25,26] and both cholinergic muscarinic and nicotinic binding sites have been demonstrated in the spinal dorsal horn[27,28] The origin of ChAT terminals has been suggested to be from local spinal cholinergic interneuron and/or descending pathways from supraspinal structures.[29]

Electrophysiological studies have demonstrated that cholinergic receptor agonists produce inhibitory effects on spinal dorsal horn neurons, including spinothalamic tract neurons.[30,31] This suggests that a spinal cholinergic system plays an important inhibitory role in the modulation of nociceptive transmission. Pharmacological studies in ‘awake’ rats have found that this spinal cholinergic inhibition is tonically active and is mediated by spinal muscarinic, but not nicotinic receptors.[32]

Since nitric oxide (NO) was shown to be a central neurotransmitter,[33,34] there have been several reports of the relationship between NO and pain processing in the brain and the spinal cord.[5,6] It is widely accepted that NO may occupy a key position in the antinociceptive and in the endogenous mediation of pain. Acetylcholine and morphine induce analgesia via activation of the arginine-NO-cGMP pathway.[11,12] Guanylate cyclase activity in the brain is markedly stimulated by NO, generated from L-arginine or provided through an exogenous source,[4] as in the present study through transdermal nitroglycerine. Evidence exists that NO modulates the synaptic transfer of signals in both the central and the peripheral nervous system.[35] The transdermal nitroglycerine patch has been related to NO formation during degradation of organic nitrates.[36] In accordance to animal[37] and clinical research,[19] NO generators did not result in analgesia. Nevertheless, a current study provides evidence that acetylcholine stimulate nitric oxide synthesis in the spinal cord,[38] and this synthesis is necessary for the expression of analgesia secondary to the cholinomimetic agent,[39] such as spinal neostigmine.

In addition, the activation of descending pain pathways involves the participation of nitric oxide, which mechanisms of action are likely to include activation of second messengers such as cyclic guanosine monophosphate (cGMP).[32] Wide-dynamic-range neurons in the superficial dorsal horn and high-threshold cells in the superficial or deep layers show reduced response after exposure to cyclic guanosine monophosphate.[40] Therefore, analgesia would be a result of predominant analgesic action on superficial spinal layers.

Anatomic evidence also supports the connection between NO and acetylcholine. As explained earlier, ChAT-positive terminals are found in the spinal dorsal horn and both cholinergic muscarinic and nicotinic binding sites have been demonstrated in the spinal dorsal horn. Recent studies show that Nitric Oxide Synthase (NOS) contain neurons located in Laminae I through III of the dorsal horn[41] (the superficial dorsal horn and the intermediolateral cell column regions of the spinal cord)[42] and probably function as interneuron modulating the sensory processing[7] in the spinal cord that contain choline acetyl transferase[43]

## CONCLUSIONS

Our results show that neostigimise increases the duration of analgesia of bupivicaine and transdermal nitroglycerine increases this postoperative analgesia further, though nitroglycerine itself does not show any analgesic potential of its own.
